This article has been retracted.

# The structure of SV40 large T hexameric helicase in complex with AT-rich origin DNA

**DOI:** 10.7554/eLife.18129

**Published:** 2016-12-06

**Authors:** Dahai Gai, Damian Wang, Shu-Xing Li, Xiaojiang S Chen

**Affiliations:** 1 Departments of Biological Sciences and Chemistry, Molecular and Computational Biology Program, University of Southern California, Los Angeles, United States; 2 Department of Biological Sciences, Genetic, Molecular and Cellular Biology Program, Keck School of Medicine, University of Southern California, Los Angeles, United States; 3 Center of Excellence in NanoBiophysics, University of Southern California, Los Angeles, United States; 4 Norris Comprehensive Cancer Center, University of Southern California, Los Angeles, United States; Howard Hughes Medical Institute, Massachusetts Institute of Technology, United States

**Keywords:** structural biology, DNA replication, APOBEC deaminase, *E. coli*, Human, Virus

## Abstract

DNA replication is a fundamental biological process. The initial step in eukaryotic DNA replication is the assembly of the pre-initiation complex, including the formation of two head-to-head hexameric helicases around the replication origin. How these hexameric helicases interact with their origin dsDNA remains unknown. Here, we report the co-crystal structure of the SV40 Large-T Antigen (LT) hexameric helicase bound to its origin dsDNA. The structure shows that the six subunits form a near-planar ring that interacts with the origin, so that each subunit makes unique contacts with the DNA. The origin dsDNA inside the narrower AAA+ domain channel shows partial melting due to the compression of the two phosphate backbones, forcing Watson-Crick base-pairs within the duplex to flip outward. This structure provides the first snapshot of a hexameric helicase binding to origin dsDNA, and suggests a possible mechanism of origin melting by LT during SV40 replication in eukaryotic cells.

**DOI:** http://dx.doi.org/10.7554/eLife.18129.001

## eLife digest

When a cell divides to form a new cell, it must also copy its DNA. An important step for starting DNA replication is to break or “melt” the bonds between the two strands of DNA that make up the double helix. This happens at a specific site on the DNA called the replication origin, and allows double-stranded DNA to partially unwind into two single strands. Each strand acts as a template to form a new copy of its partner strand.

In many organisms, ring-shaped proteins called helicases attach directly to double-stranded DNA to melt the bonds at the replication origin. Viruses also have helicases that they can use to hijack the cell’s replication machinery and get it to copy the viral DNA. One such helicase called Large T antigen is an important part of a tumor virus called simian virus 40. Large T has a ‘hexameric’ structure, similar to the cell’s own helicases, and researchers often use it as a model for studying the replication process. However, key questions remain. How do hexameric helicases interact with the double-stranded DNA replication origin? And what are the molecular mechanisms by which these helicases melt bonds in double-stranded DNA?

Gai et al. used a technique called X-ray crystallography to examine the molecular structure of the Large T helicase when it is attached to DNA. The resulting structures show that six subunits of Large T helicase assemble a ring around the replication origin, each making unique bonds with the DNA. The helicase ring squeezes the DNA, partially breaking the bonds between the DNA strands and causing local melting of the DNA.

With the understanding of how the Large T hexamer helicase interacts with its DNA replication origin and how its assembly initiates DNA melting, the future challenge is to explain the process by which the partially melted origin opens up fully for replication to begin.

**DOI:** http://dx.doi.org/10.7554/eLife.18129.002

## Introduction

DNA replication is essential in the inheritance of genetic information for living organisms. The initiation of DNA replication involves crucial steps in the assembly of replication proteins at the origin and in the subsequent melting of the origin DNA. For DNA replication in prokaryotic cells, the initiator protein, DnaA, first binds to the replication origin to initiate origin melting. The replicative DnaB-family of hexameric helicases are then loaded onto the fully melted single-stranded DNA (ssDNA) for replication fork unwinding [reviewed in O'Donnell et al. (2013)] and references therein). For DNA replication in archaeal and eukaryotic cells, replicative helicases, such as minichromosome maintenance proteins (MCM) and SV40 Large T Antigen (LT), load onto the origin dsDNA as head-head (or N-N) double hexamers [reviewed in Fanning and Zhao (2009); Gai et al. (2010); O'Donnell et al. (2013); Slaymaker and Chen (2012) and references therein]. The origin bound by the double hexameric helicases, together with other replication factors, will eventually melt the duplex and produce a pair of replication forks. Despite extensive efforts, the molecular interactions of these hexamer helicases in archaeal and eukaryotic replication systems with their origin dsDNA have yet to be defined.

In SV40 DNA replication, the host eukaryotic cellular replication machinery is utilized, except for the MCM helicase, whose function is fulfilled by SV40 LT. As a result, the SV40 replication system serves as a model for studying the eukaryotic replication process [reviewed by Bullock and Simmons (1997); Fanning and Zhao (2009) and references therein]. To initiate DNA replication, MCM helicase proteins from archaeal and eukaryotic cells assemble a double hexamer at the origin dsDNA (Evrin et al., 2009; Fletcher et al., 2003; Mendez and Stillman, 2003; Remus et al., 2009; Ticau et al., 2015), a process that requires the cellular origin recognition complex (Orc) as well as additional protein factors. By contrast, the SV40 LT helicase alone is sufficient in recognizing its origin and assembles as a double hexamer at the origin dsDNA (Borowiec et al., 1990; Cuesta et al., 2010; Valle et al., 2006). On linear blunt-ended dsDNA, containing the SV40 origin sequence, purified LT alone can generate bi-directional unwinding forks from the dsDNA origin region, producing 'rabbit ear'-like single-stranded DNA loops emanating out of the LT complex (Wessel et al., 1992b). These studies, together with other reports (Borowiec et al., 1990; Borowiec and Hurwitz, 1988; Joo et al., 1998; Kim et al., 1999; Valle et al., 2006), demonstrate that LT alone can sufficiently assemble as a double hexamer at the origin, melt the origin DNA, and generate bi-directional unwinding forks. Previous biochemical studies also demonstrate that assembly of the LT double hexamer on the origin dsDNA leads to local melting around the AT-rich sequences (Borowiec et al., 1990; Borowiec and Hurwitz, 1988). Available structural and biochemical data suggest that the melted DNA region is located within the AAA+ domain of LT (Kumar et al., 2007; Shen et al., 2005).

LT has three major functional domains (Figure 1A): the Dna-J homology domain, the origin-binding domain (OBD), and the helicase domain (Bullock, 1997; Gai et al., 2004a). LT helicase domain consists of a Zn-domain and an AAA+ (ATPases Associated with diverse cellular Activities) domain (Figure 1A). The AAA+ domain has a fold of five β-strands at its core, with a few helices that function as a motor domain by coupling the energy of ATP binding and hydrolysis (Neuwald et al., 1999; Ogura and Wilkinson, 2001). The core replication origin DNA of SV40 consists of 64 base pairs (bps) (Figure 1B) that can be divided into two halves, the AT-half and the early palindrome half (EP-half), each containing two GAGGC penta-nucleotide sequences (PEN) plus a stretch of AT-rich sequence (Dean et al., 1987; Deb et al., 1986; Sreekumar et al., 2001). An individual OBD alone has been shown to bind specifically to the PEN sequences (Bochkareva et al., 2006; Deb et al., 1987; Meinke et al., 2007, 2011, 2014). However, when the LT construct containing the OBD-helicase domain in one polypeptide (residues 131–627 or LT131) is used, the OBD (residues 131–258) binds to a GC pseudo-PEN site in addition to the canonical PEN, and the AAA+ domain of the helicase binds to the AT-rich sequences of the origin (Chang et al., 2013). Both the AT-half and EP-half of the origin can support the assembly of one LT hexamer (Joo et al., 1998; Kim et al., 1999; Shen et al., 2005), and a full core origin supports the formation of two hexamers arranged in an N-to-N configuration (Bullock et al., 1997; Cuesta et al., 2010; Valle et al., 2006).

**Figure 1.** SV40 LT domain structure, core origin DNA (oriDNA), and the co-crystal structure of the LT helicase domain bound to the AT-half oriDNA. (**A**) LT domain organization (drawn to scale), with the LT131 used for the co-crystallization study indicated at the top. (**B**) The full 64-bp core replication oriDNA of SV40. The four penta-nucleotides (PEN) (GAGGC (in red)) are flanked in the AT-half and in the EP-half origin. The AT-half origin DNA (boxed in blue) is co-crystallized with the LT hexameric helicase in this study. (**C**) The gel filtration profile (Superose 6) of LT131 alone or in complex with the AT-half oriDNA in the presence of ADP or ATP without Mg^2+^. LT131 alone equilibrates between hexamer and monomer peaks (red), but will form a stable hexamer when ATP is present (Gai et al., 2004a; Li et al., 2003). In the presence of ATP (blue) or ADP (green), LT131 forms stable hexamer-DNA complexes with the 32-bp AT-half oriDNA, which migrate slightly larger than the LT131 hexamer alone. The LT-oriDNA-ATP complex isolated from this peak showed no obvious dissociation after up to six hours, suggesting a very stable complex without ATP hydrolysis. (**D**, **E**) The preformed LT hexamer-oriDNA complexes (made by first incubating LT131 with oriDNA and ATP, then adding Mg^2+^ last to initiate unwinding, see Materials and methods) is active in unwinding the oriDNA (**D**). For comparison, (**E**) shows the unwinding results obtained using LT131 with no preformed (un-preformed) hexamer-oriDNA complexes (made by adding LT131 and Mg^2+^ last to initiate unwinding, see Materials and methods);this shows unwinding efficiency similar to that obtained using the preformed LT-oriDNA complex (**D**). This result suggests that the preformed stable LT-oriDNA complex is active in unwinding the oriDNA. Note that the unwound ssDNA product migrates slower than the dsDNA substrate because of hairpin formation at the palindrome origin sequence. (**F**) Overall view of the LT hexameric helicase bound to the AT-half origin DNA (32 bp) in the central channel. (**G**) Superimposition of the DNA-free (green) and DNA-bound (orange) hexamer structures, both of which are in an ADP-bound state. For clarity, only two subunits of hexamer are shown so that it is possible to visualize the β-hairpins and DRF loops. The Zn-domain and the AAA+ domain of LT are indicated. **DOI:** http://dx.doi.org/10.7554/eLife.18129.003

**Figure 1—figure supplement 1.** Comparing the DNA register in the dimeric LT structure bound to the EP-half origin with that in the hexameric LT structure bound to the AT-half origin DNA. (**A**) The 64-bp full core origin of SV40. The EP-half and AT-half origins are indicated. For the EP-half origin, the sequence that is in contact with OBD1, OBD2, and the helicase domain of the LT131 dimer, as revealed in the LT131 dimer-DNA co-crystal structure (PDBid: 4GDF), is indicated. For the AT-half origin, the sequence that is in contact with LT helicase domain, as revealed in the LT helicase hexamer-DNA co-crystal structure, is indicated. (**B**) LT131 dimer-DNA co-crystal structure, showing how the two LT subunits bind to EP-half origin DNA (PDBid: 4GDF). The EP-half origin sequence is positioned next to the complex structure with the same DNA register to indicate the corresponding DNA sequence bound by the different domains of LT131. With OBD1 binding to PEN1, OBD2 cannot reach PEN2 from subunit 2 because the linker is not long enough. Instead, OBD2 binds to pseudo-PEN1, with an 180° rotation from OBD1. (**C**) The LT helicase hexamer-DNA co-crystal structure, with the AT-half origin sequences positioned next to the complex structure with the same DNA register to indicate the corresponding DNA sequences bound by LT. For comparison, we tried to best align the register of bound DNA in this panel with that in (**B**). The PEN1’ and pseudo-PEN’ positions are indicated. **DOI:** http://dx.doi.org/10.7554/eLife.18129.004

**Figure 1—figure supplement 2.** The full occupancy of ADP at all six nucleotide pockets of an LT hexamer and the arrangement of the β-hairpins (β-HP) and DRF loops of the AAA+ domain. (**A**) Omit map of ADP density from an LT hexamer-DNA complex structure (one asymmetric unit), showing strong density of the ADP (drawn at 5 sigma level) at all six sites. Even though the electron densities for the six sites are not identical, they are all strong, indicating full occupancy in the DNA-bound hexamer structure, as is the case in all previously determined DNA-free LT hexamer structures. (**B**) A close-up view at one of the ADP densities, drawn at sigma contour level 5. (**C**) The β-hairpins (β-HP) and DRF loops of the AAA+ domain in the central channel of a LT hexamer. The β-hairpin residues K512/H513 and the DRF residues D455, R456, F459 are shown as sticks. For clarity, only two opposing subunits of the hexamer are drawn. (**D**) The near-planar arrangement of the six β-hairpins (β-HP) and DRF loops in the AAA+ domain of the LT hexamer in the DNA complex structure, showing that the β-hairpins and loops are not absolutely planar, but slightly offset. The H513 on the β-hairpin tip is drawn in sticks. **DOI:** http://dx.doi.org/10.7554/eLife.18129.005

In order to understand how the LT hexameric helicase assembles at the origin and interacts with the origin DNA, we determined the structure of a LT hexameric helicase in complex with the AT-half of the origin to a resolution of 2.9 Å. This co-crystal structure, the first for a hexameric helicase bound to its origin dsDNA in its central channel, reveals detailed molecular interactions between the six subunits and the origin sequence. In addition, the structure also shows that a stretch of the AT-rich sequence bound within the narrow channel of the AAA+ domain is partially melted, most likely as a result of a 'squeezing' of the two phosphate backbones by the assembled hexameric helicase, which may be assisted by the specific interactions between residues of the LT AAA+ domain and the AT-rich origin sequence. The structural data reported here offer a mechanistic explanation for how LT accomplishes initial origin melting and may have implications for other related eukaryotic replicons.

## Results

### LT deletion constructs capable of unwinding origin-containing dsDNA

In order to study the replicative helicase assembly around the origin DNA for SV40 replication initiation, we used an SV40 LT construct LT131-627 (residues 131–627, referred to as LT131 hereafter) — which includes the OBD domain (residues 131–258) and the helicase domain (residues 260–627) (Figure 1A) — for co-crystallization with the AT-half or the EP-half of the origin dsDNA (Figure 1B). Previously, using electron microscopy (EM), we showed that a slightly longer LT108 construct can assemble as a double hexamer on dsDNA containing the full 64-bp core origin in the presence of ATP or ADP, and can support the replication of such DNA in HeLa cell extract (Cuesta et al., 2010). To the best of our knowledge, LT is unique in that it can unwind blunt-ended dsDNA containing its origin sequence, whereas the other hexameric helicases characterized to date are not capable of unwinding blunt-ended dsDNA efficiently without the aid of additional protein component(s). We previously also showed that purified LT131 alone, like the full-length LT, can efficiently unwind blunt-ended dsDNA containing the origin sequences in vitro (Chang et al., 2013). LT131 also forms stable hexameric complexes bound to the 32-bp AT-half of the origin along with ADP or ATP (Figure 1C). Interestingly, these stable pre-formed hexamers/double hexamers on origin dsDNA are also capable of unwinding the DNA when Mg^2+^ is supplied (Figure 1D,E), which is consistent with previous reports for full-length LT (Uhlmann-Schiffler et al., 2002). This result suggests that the LT double hexamers assembled at the origin sequence are fully competent in generating the initial local origin melting to promote the complete unwinding of the dsDNA.

### Overall structure of the LT-dsDNA complex

We obtained co-crystals of the complex containing LT131 (Figure 1A) and the 32-bp AT-half origin dsDNA (bps 1–32, plus 3’-T overhangs, Figure 1B) in the presence of ADP and Mg^2+^, and determined the structure to a resolution of 2.9 Å (Table 1). The structure shows one hexamer of the helicase domain (residues 266–627) binding to the dsDNA in the hexamer channel in each asymmetric unit (Figure 1F). All of the 32-bp AT-half origin dsDNA sequences were built into the DNA structure (Figure 1B, Figure 1—figure supplement 1A–C). The hexamer structure contains the entire helicase domain (Figure 1A), without the N-terminal OBD (residues 131–265) built into the model. The OBDs are actually visible as six blobs of smeared electron density located N-terminal to the Zn domain, suggesting disordered OBDs, possibly due to the lack of interactions between any of the six OBDs with the PEN or pseudo-PEN origin sequences after the completion of the hexamer assembly. This is clearly different from the previously reported co-crystal structure of the dimeric LT131 in complex with the EP-half of the origin sequence (Chang et al., 2013), in which one of the two OBDs binds to the canonical PEN in the same way that has been reported by others (Bochkareva et al., 2006; Meinke et al., 2007), and the other OBD binds to a newly identified pseudo-PEN (GC) sequence (Figure 1—figure supplement 1B).

**Table 1.** Crystallographic data and refinement statistics. **DOI:** http://dx.doi.org/10.7554/eLife.18129.006

	Co-crystal of complex containing LT131, AT-half origin dsDNA, and ADP
**Data collection**	
Space group	P1
Wavelength (λ)	1.1159 (Å)
Cell: *a, b, c* (Å)	107.485, 107.587, 107.870
Angles: α, β, γ (°)	107.133, 106.954, 106.865
Resolution (Å)	50–2.90 (2.95–2.90)
*R*_merge_ (%)	5.3 (79.7)
*I* / σ*I*	28.9 (1.52)
Completeness (%)	97.7 (89.1)
Redundancy	3.1 (2.5)
Refinement	
Resolution (Å)	50.0–2.9
Unique reflections	85, 533
*R*_work_ / *R*_free_ (%)	27.8/30.4
No.atoms	
Protein	17,598
DNA	1354
Ion	6
ADP	162
**r.m.s deviations**	
Bond lengths (Å)	0.007
Bond angles (°)	1.194

*Highest-resolution shell is shown in parentheses.

All six nucleotide pockets of the LT hexamer are fully occupied by ADP, as shown by the strong electron density at all six pockets (Figure 1—figure supplement 2A–B), which is consistent with the all-or-none nucleotide binding-mode on all the previously determined hexamer structures of LT (Gai et al., 2004b). This DNA-bound hexamer essentially adopts the same structure as the previously determined DNA-free ADP-bound hexamer (Gai et al., 2004b), with an Cα r.m.s deviation of superposition around 0.79 (Figure 1G). Similar to all the DNA-free hexamer structures of the LT helicase domain (Gai et al., 2004b; Li et al., 2003; Lilyestrom et al., 2006; Zhou et al., 2012), the DNA-bound hexamer reveals that the six subunits are arranged with only minor offset to break symmetry (Figure 1—figure supplement 2C,D), which can be considered to be a near-planar ring (referred to as a planar ring hereafter for convenience). Within the AAA+ domain of LT, there is a β-hairpin bearing a H513 residue on the inner surface of the hexamer channel (Figure 1—figure supplement 2C), and the β-hairpin displays movement of more than **17 Å **along the channel during conformational changes triggered by ATP binding/hydrolysis and release (Gai et al., 2004b). C-terminal to the β-hairpin is the DRF loop that carries residues D455, R456, F459 (DRF) pointing into the channel (Figure 1—figure supplement 2C). In the planar ring structure of the LT hexamer, the six β-hairpins and the DRF loops form a narrowest channel segment around the bound dsDNA (Figure 1—figure supplement 2D).

**Figure 2.** The structure of the LT hexamer helicase in complex with the AT-half origin. (**A**) The AT-half origin DNA sequence contains 32 bp with 3’-T overhangs bound by LT hexameric helicase in (**B**). The side-bars indicate the DNA contacts by different regions within the LT helicase channel, including the Zn-domain, the central chamber, the β-hairpins (β-HP) and DRF loops (DRF-LP). PEN1’ and pseudo-PEN1’ are not occupied by OBD in LT hexamer structure. The deformed region is indicated on the side. (**B**) The structure of LT131 hexamer bound to the 32-bp AT-half origin DNA. For clarity, only two subunits (one on each side) are shown. The positions of the PEN1’ and pseudo-PEN1’ where OBD1 and OBD2 would bind are indicated. (**C**) The structure of LT131 dimer bound to the 32-bp EP-half origin DNA (PDBid: 4GDF), showing one of the two subunits using its OBD to bind PEN1. The pseudo-PEN1’ is bound by the OBD of the second subunit of the dimer (Figure 1—figure supplement 1A,B); thehelicase domain of the dimer, including the Zn-domain and the AAA+ domain, binds to the AT-rich region of the EP-half origin. The structures in (**B**) and (**C**) are drawn to scale and aligned side-by-side for comparison between the hexamer-DNA and dimer-DNA complexes. (**D**) The dsDNA segment bound in the AAA+ channel is deformed and locally melted. (**E**) Top view of the LT hexamer (each subunit in a discrete color) from the N-terminal end, showing dsDNA in the central channel. **DOI:** http://dx.doi.org/10.7554/eLife.18129.007

**Figure 2—figure supplement 1.** Initial unbiased electron density inside the hexameric channel, and DNA orientation and register confirmed by Bromo-labeled dC (Br-dC) DNA. (**A**) A section of the initial electron density map, which was calculated on the basis of the MR LT hexamer model alone prior to any DNA building, showing the dsDNA density with clear nucleotide base steps running through the central channel. The map was calculated as follows (also described in the Materials and methods session). The MR solution model of the LT hexamer was partially deleted on the β-hairpin and DRF loop residues facing the central channel to avoid model bias for the residues that potentially interact with DNA in the channel. The partially deleted MR LT hexamer model was used for calculations of the initial phases and for mask calculation for NCS averaging. Two-domain six-fold NCS averaging was then performed, using a tight mask so that a large central channel space where DNA is located was masked out during NCS averaging, which will avoid averaging the DNA density out in the central channel. The resulting NCS averaged map was drawn here at sigma level 1, which shows the clear DNA base steps in the central channel. (**B**, **C**) The AT-half origin DNA inside the hexamer channel (**B**), and the corresponding DNA sequence (**C**), with the Bromo-labeled dC (Br-dC at position 12) indicated (colored in green). (**D**, **E**) Difference Fourier map of the anomalous data collected from the LT-DNA co-crystals containing the Bromo-labeled dC (Br-dC) DNA at the 12th dC position as shown in (**C**). The map was drawn with contour sigma level 2.0, showing a strong peak (viewing from two angles) at the expected location for the labeled dC, confirming the DNA orientation and register in the hexamer channel. **DOI:** http://dx.doi.org/10.7554/eLife.18129.008

### DNA structure inside the hexamer channel

The entire AT-half origin dsDNA sequence built into the hexamer channel of LT is shown in Figure 2A and B (also Figure 1—figure supplement 1), with one LT subunit bound to the 32-bp EP-half origin taken from the LT131 dimer-dsDNA structure shown in Figure 2C for comparison (see Figure 1—figure supplement 1B for the dimer structure). The DNA orientation and register is further verified by using Bromo-labeled dC (Br-dC) DNA in the co-crystal structure (Figure 2—figure supplement 1). Bps 1–15 of the origin dsDNA are located outside the channel; bps 6–23 are within the Zn-domain channel; bps 24–26 are in the central chamber (a wide chamber); and bps 27–32 are within the AAA+ channel (Figure 2A). The dsDNA segment bps 1–24 is in B-form, while a stretch of A-T base pairs, most of which are within the AAA+ channel lined by the β-hairpins and DRF loops, is severely deformed (bps 25–32, Figure 2A,B,D), disrupting the base paring to yield locally melted duplex DNA. The narrow parts of the hexamer channel in the AAA+ domain, lined by the β-hairpins and DRF loops, is between 14–19 Å (Figure 1G), which is narrower than the diameter of the B-form DNA. The B-form DNA segment has approximately 19–20 Å distances between its two phosphate backbones. However, the backbone distances in the deformed DNA segment (bps 25–32) are mostly in the range of 15–16 Å. The minor groove within this deformed stretch hasbackbone distances of around 4.5–5.0 Å, also much narrower than that of the B-form DNA segment, whichhas the distances around 7.2–10.0 Å. One major consequence of the closer phosphate backbone distance within the stretch of deformed DNA is the disruption of normal Watson-Crick base-paring within the duplex (Figure 2D). Below, we describe the detailed structural features and the protein-DNA interactions along the central channel in the N- to C- direction.

### dsDNA interactions with the N-terminal Zn-domain

The LT hexamer channel around the N-terminal Zn-domain has an opening of approximately 21 Å between the side chains at its narrowest point, which widens greatly towards the central chamber. The entire channel length from the Zn-domain to the C-terminal DRF-loop is approximately 60 Å (Figure 1G), encompassing a total of 17 bps of oriDNA bound within the helicase channel (Figure 2A,B). The Zn-domain channel interacts with 8 bps of this oriDNA, all through the phosphate backbones of the DNA.

Within the Zn-domain region, the dsDNA is in B-form and fits through the channel tightly, with its two phosphate backbones interacting with charged or polar amino acids in the channel surface (Figure 3A–F). Interestingly, each of the two DNA backbones interact with nearly identical sets of amino acid residues (N267, K331, N332, K334 and T335) that come from different subunits (subunits i-vi) and that are arranged in different orientations (Figure 3C–F, Supplementary file 1). Specifically, the 5’→3’ ssDNA interacts with a set of residues from N→C domain of the helicase containing: N267 of subunit i and ii, K331 of i, ii, and iii, N332 of ii, iii, and iv, and T335 of iv and v (Figure 3C–D). Its complementary strand (also from 5’→3’ direction), interacts with a similar set of residues but from different subunits: K334 of i and ii, T335 of i and vi, N332 of v and vi, and N332 and K331 of v (Figure 3E–F). Therefore, despite their opposite orientations, the two antiparallel ssDNA strands of the B-form DNA interact with two different sets of but chemically identical, amino acids along the channel surface of the Zn-domain. In other words, these two sets of amino acid residues make near identical bond interactions with DNA phosphate backbones running in either the 5’→3’ or 3’→5’ orientation.

**Figure 3.** Detailed interactions of origin DNA with the Zn-domain of LT. (**A**, **B**) Two different views of dsDNA inside the LT hexameric channel, one with two complete subunits out of six (**A**) and the other with the DNA-binding residues on the Zn and AAA+ domains of all six subunits (**B**). (**C**, **D**) Two views tshowing the detailed interactions of the 5’→3’ DNA strand with LT residues inside the Z-domain channel from the N→C direction. The six subunits are labeled as i, ii, iii, iv, v, vi. The residues contacting the DNA are shown as sticks. (**E**, **F**) Two views showing the detailed interactions of the 3’→5’ DNA strand with LT residues inside the Z-domain channel from the N→C direction. **DOI:** http://dx.doi.org/10.7554/eLife.18129.009

### dsDNA interactions with the C-terminal AAA+ domain

The central channel narrows down to a much smaller opening at the AAA+ domain where the β-hairpins and the DRF loops are arranged in near-planar rings (Figure 1D, Figure 4—figure supplement 1A). The channel segment composed of β-hairpins and the DRF loops is approximately 22 Å in length, and binds 6 bps of deformed dsDNA (bps 27–32, plus the 3’-T overhang, Figure 2A). The planar arrangement of the β-hairpins and DRF loops of LT observed in this dsDNA-bound structure and the previously reported apo-structures (Gai et al., 2004b; Li et al., 2003; Lilyestrom et al., 2006; Zhou et al., 2012)(Figure 4—figure supplement 1A,B) are in sharp contrast to the staircase β-hairpins reported for the E1 helicase in the ssDNA-bound (Enemark and Joshua-Tor, 2006) and apo-structure (Sanders et al., 2007) (Figure 4—figure supplement 1C–D). In the ssDNA-bound E1 structure, each of the six spirally arranged β-hairpins of the E1 hexamer has similar interactions with a spirally shaped six-nucleotide oligo-dT via the phosphate backbones of the ssDNA (Figure 4—figure supplement 1C).

The planar arrangement of the six β-hairpins and DRF loops in the dsDNA-bound hexamer structure of LT is nearly identical to that in the DNA-free LT hexamer structure, including the channel openings and the conformations of the β-hairpins and DRF loops (Figure 1G). Because this stretch of channel is clearly narrower than the dimension of B-form dsDNA, the dsDNA bound inside has to be deformed in order to fit through the smaller channel. As a result, the two backbones in this segment are closer to each other than in standard B-form dsDNA; this deformation is a consequence of compression by two opposing subunits of the hexamer around the narrow channel. The deformation of DNA should also be assisted by its interactions with residues on the β-hairpins and DRF loops in the channel walls (Figure 4A–F). When the two phosphate backbones are compressed by the β-hairpins and the DRF loops, the base-pairs within the duplex are forced to flip outward, leading to the local melting of the dsDNA (Figure 4A–F).

**Figure 4.** Detailed interactions of origin DNA with the AAA+ domain. (**A**, **C**, **E**) Detailed interactions of DNA with three pairs of subunits within the LT hexamer: subunit pair **i** & **iv** (**A**), **ii** & **v** (**C**), and **iii** & **vi** (**E**). The β-hairpin residues K512/H513 and DRF loop residues D455/R456/F459 that bind to the DNA are labeled. (**B**, **D**, **F**) The detailed interactions of the oriDNA with the same three pairs of LT subunits shown in (**A**) [matching **B**], (**C**) [matching **D**], and (**E**) [matching **F**]. Dashed lines indicate hydrogen-bond interactions between LT residues and DNA (in the stick model). Some of LT residues are 5–7 Å away from DNA, and would be suitable for the water-mediated formation of hydrogen bonding. In addition, a number of LT residues are within Van der Waals distance of the bound DNA, forming hydrophobic packing interactions; these residues include K512 of subunit **i** (**i**-K512), **i**-F459, **iv**-F459, **ii**-F459, **v**-F459, **vi**-F459, and **vi**-H513. The dislocated bases in the disrupted bases-pairs (in the partially melted DNA region) are drawn in thick sticks, with the DNA sequences of this region shown to the left of panel **B**. The structure shows clearly that identical residues on different subunits make unique contacts with the phosphate backbones and the major or minor gr oves of the DNA; this is possible due to the near-planar arrangement of the six subunits. **DOI:** http://dx.doi.org/10.7554/eLife.18129.010

**Figure 4—figure supplement 1.** The planar and staircase arrangements of β-hairpins in the hexamer structures of LT and E1. (**A**) The near-planar arrangement of the six β-hairpins (indicated by an arrow) in the hexamer channel of LT. Such near-planar arrangement is maintained in all the structures of LT hexamer determined to date, regardless of their dsDNA-bound or DNA-free states. (**B**) A close-up view of the near-planar arrangement of the six LT β-hairpins from (**A**), with H513 on the β-hairpin tip shown in sticks. The close-up view reveals that the six H513 and β-hairpins have no real six-fold symmetry. However, a near-planar arrangement is obvious when compared with the staircase arrangement shown in (C). (**C**) The staircase arrangement of the six β-hairpins (and the tip His residue) in the E1 hexameric channel, showing a six-nucleotide ssDNA (in thin sticks) with each of the six nucleotides havingsimilar interactions with the six β-hairpins (PDBid: 2GXA). (**D**) Alignment of the β-hairpins in the central channel of E1 hexamer structures in the ssDNA-bound state (PDBid: 2GXA, in green) and the DNA-free state (PDBid: 2V9P, in orange), showing the same staircase arrangement for the β-hairpins, regardless of ssDNA-bound or ssDNA-free state. **DOI:** http://dx.doi.org/10.7554/eLife.18129.011

The major residues interacting with dsDNA in the AAA+ domain include K512 and H513 on the β-hairpins, and residues D455, R456, and F459 (DRF) on the DRF loops (Figure 4). All six subunits use these same residues to interact with DNA, but on each subunit, these residues contact DNA differently as a consequence of the near-planar arrangement of the β-hairpins and DRF loops (Figure 4B, D, F). The β-hairpin residues K512/H513 from the subunit pairs ii + v (Figure 4C,D) and iii + vi (Figure 4E,F) more or less impinge on the two DNA backbones from opposite sides, while the DRF loop residues D455/R456/F459 from the subunit pairs i + iv (Figure 4A,B) and ii + v (Figure 4C,D) act on the phosphate backbones similarly, pushing the two phosphate backbones within this region closer to each other. This may be sufficient to destabilize the Watson-Crick base-pairing, forcing the bases to flip outward. Thus, these amino acids on the β-hairpins and DRF-loops from different LT subunits interact with the deformed DNA from the major and minor grooves as well as the phosphate backbones (Figure 4A–F, Supplementary file 2).

**Table 2.** The central channel dimensions at the β-hairpins and DRF loops in the hexamer structures of various nucleotide-bound states determined previously and in the DNA-bound state reported here. **DOI:** http://dx.doi.org/10.7554/eLife.18129.012

	Between β-hairpin tip residues K512 and H513 (Å)	Between DRF loop tip residues D455 and R456 (Å)
		
dsDNA-bound ADP-hexamer (this report)	19.5, 19.9, 20.1	14.8, 14.8, 15.0
dsDNA-free ADP-hexamer (PDB:1SVL)	11.6, 13.1, 14.6	14.0, 16.0, 18.3
dsDNA-free ATP-hexamer (PDB:1SVM)	6.90, 7.40, 8.90	7.90, 8.30, 8.30
dsDNA-free Empty hexamer (PDB:1N25)	14.5	17.9

## Discussion

Hexameric helicases in prokaryotic DNA replication are loaded onto ssDNA generated at the origin by the action of DnaA [reviewed by O'Donnell et al. (2013)] and references therein), whereashelicases in eukaryotic DNA replication systems (such as MCM and SV40 LT) form a double hexamer at the replication origin dsDNA, which must be melted in order to propagate fully opened bi-directional forks (Borowiec and Hurwitz, 1988; Evrin et al., 2009; Hurwitz et al., 1990; Remus et al., 2009; Ticau et al., 2015; Valle et al., 2006; Wessel et al., 1992a). How eukaryotic origin dsDNA is melted by the hexamer/double hexamer helicase is unclear. Here, we reported a co-crystal structure of an ADP-bound LT hexameric helicase with a 32-bp AT-rich origin dsDNA inside its central channel. The structure reveals detailed molecular interactions of the hexameric helicase with the origin DNA sequence within the hexamer channel. While the majority of the origin dsDNA in the larger N-terminal portion of LT hexamer is in B-form, the AT-rich sequence bound within the narrow AAA+ channel segment is partially melted, revealing a probable origin-melting mechanism.

### Comparing the dsDNA-bound and DNA-free apo-structures of the LT hexamer

Interestingly, the DNA-bound and DNA-free forms of the LT hexameric helicase structures are largely the same. This includes both the small opening of the hexamer channel in the AAA+ domain and the near-planar arrangement of the six subunits, β-hairpins, and DRF loops in the central channel. Several DNA-free hexameric structures of the LT helicase domain have been reported previously, including the structures of three different nucleotide (nt)-bound states: the empty form alone or in complex with other proteins (Li et al., 2003; Lilyestrom et al., 2006; Zhou et al., 2012); the ADP-form, with all six nt pockets occupied by ADP, and the ATP-form, with all six nt pockets occupied by ADP-BeF_3_^-^ (Gai et al., 2004b). These different DNA-free hexameric structures reveal substantial concerted conformational changes for the six β-hairpins and DRF loops within and along the central channel of LT hexamer, but the overall conformations of these hexamers are quite similar (Gai et al., 2004b; Li et al., 2003; Lilyestrom et al., 2006; Zhou et al., 2012). Subsequent comparisons of the dsDNA-bound and DNA-free LT hexameric helicase structures, both in the ADP-form, show that these structural features are essentially maintained regardless of DNA binding. This strongly suggests that the binding of dsDNA in the central channel, per se, has no major impact on the overall conformation of the protein hexamer. Obviously, it is the conformational state of the protein hexamer that determines the conformation of the bound dsDNA. By extension, the cyclic conformational changes of hexameric LT are expected to drive the remodeling of the bound dsDNA, as shown by the different nt-bound states: ATP-binding shrinks the central channel further than ADP-binding and triggers large β-hairpin movement inside the central channel (Gai et al., 2004b).

By contrast, even though the E1 hexameric helicase shows a staircase arrangement of the six β-hairpins instead of a planar arrangement, the staircase conformation is observed in the E1 ssDNA-free structure and further maintained in the E1 ssDNA-bound structure. This evidence provides another example of how protein conformations in the DNA-free form may provide insight into how these proteins interact with DNA (Figure 4—figure supplement 1C–D) (Enemark and Joshua-Tor, 2006; Sanders et al., 2007). Interestingly, the co-crystal structures of the prokaryotic helicase DnaB and the Rho RNA translocase, in complex with ssDNA and ssRNA, respectively, also reveal a spiral-like arrangement of their entire six subunits (Itsathitphaisarn et al., 2012; Thomsen and Berger, 2009), suggesting that these hexameric helicases/translocases may bind single-stranded nucleic acids using a spiral arrangement.

How then, are we able to reconcile the near-planar conformation of the β-hairpins observed in the LT hexameric helicase with the staircase conformations observed in E1 and other hexameric helicases? One simple explanation could be that planar β-hairpins in the LT-dsDNA structure and staircase β-hairpins in the E1-ssDNA structure represent two distinct stages of DNA replication. The LT-dsDNA structure may correspond to a pre-initiation hexameric complex that is assembled at the origin before it propagates into full replication forks; whereas, the E1-ssDNA structure may represent a hexameric helicase encircling a single strand of DNA for later-stage replication fork unwinding (Enemark and Joshua-Tor, 2008; Lee et al., 2014). This simple explanation would then imply an ability of LT and E1 to switch between the planar and staircase conformations, even though only one conformation has been consistently observed in structures of either protein determined to date. It is possible that the crystallographic packing somehow selectively traps the β-hairpins in the planar conformation for LT and the staircase conformation for E1, despite the crystallization buffer condition. One other major difference between E1 and LT is that E1 requires the assistance of an E2 protein for origin assembly [reviewed by McBride (2013) and references therein], whereas LT alone is sufficient for origin assembly. However, we cannot completely rule out the possibility of other potential mechanistic differences in origin assembly and origin melting by LT and by E1 helicases.

### A mechanism for origin melting: squeeze-to-open

In all determined hexameric helicase structures of LT, including the mutiple DNA-free structures reported previously (Gai et al., 2004b; Li et al., 2003; Lilyestrom et al., 2006; Zhou et al., 2012) and the dsDNA-bound structure reported here, the channel opening within the N-terminal Zn-domain remains the same, whiereas the opening of the AAA+ domain channel around the β-hairpins and DRF loops vary by between 14–19Å (Figure 1G) (Table 2). It is apparent that the helicase conformations dictate the conformation of the bound DNA inside the hexameric channel. Specifically, when the origin dsDNA is bound inside the narrower segment of the channel lined by the β-hairpins and DRF loops of LT, the two phosphate backbones will be remodeled according to the size and shape of the hexameric channel. The remodeling process involves the 'squeezing' or compressing force of the β-hairpins and DRF loops pushing the two phosphate backbones closer to each other, forcing the Watson-Crick base-pairs between the two backbones to flip outwards, leading to base-pair disruption and base flipping in the AT-rich region (Figure 4A–F). Therefore, the co-crystal structure suggests that these locally melted origin base-pairs are probably the consequence of a 'squeezing' by the narrower channel formed upon the completion of the hexamer assembly, rather than a more intuitive pulling or prying apart of the two strands. The K512/H513 residues on the β-hairpins and the D455/R456/F459 residues on the DRF loops of the AAA+ domain not only apply the 'squeezing' action to the two phosphate backbones directly, but also interact with the DNA from both the major and minor groove to generate the deformation and local melting (Figure 4A–F, Supplementary file 2).

While the hexamer-dsDNA complex structure reported here has a near-planar ring of six subunits, the possibility of changing from spiral intermediate assembly to the final planar hexamer also exists. Such conformational conversion has previously been proposed to provide energy for origin melting (Bochkareva et al., 2006; Meinke et al., 2007; Schuck and Stenlund, 2005). No spiral assembly of hexamer/double-hexamer helicases on dsDNA has been reported, but spiral assembly of hexameric helicases on ssDNA has been reported for E1, DnaB, and Rho (Enemark and Joshua-Tor, 2006; Itsathitphaisarn et al., 2012; Thomsen and Berger, 2009). In the co-crystal structure of the LT131 dimer-oriDNA intermediate assembly (Chang et al., 2013), the helicase domains of the two subunits are positioned side-by-side, whereas the two β-hairpin H513 of the dimer interact with the minor groove of the oriDNA with a partially spiral arrangement along the helical groove (Figure 5A and inset). If additional LT subunits were to be added to the dimer without changing direction, it would generate a slightly offset hexamer that resembles a lock-washer ring more closely than the closed planar hexamer structure shown in this report. If such a partial helical assembly intermediate of the helicase domain were to be converted to a closed planar hexamer upon completion of a hexamer formation, additional snapping force would be generated, facilitating origin melting in the AT-rich sequence within the narrow channel.

**Figure 5.** A model for the assembly pathway of the LT double hexamer complex on the viral origin DNA (oriDNA). (**A**) The assembly of the intermediate complex containing LT dimer bound to each half of the oriDNA, as predicted on the basis of the co-crystal structure of the LT dimer and EP-oriDNA complex (PDBid: 4GDF). The four PENs (penta-nucleotides) and the pseudo-PENs recognized by OBD are colored in red and blue. In this dimer intermediate, PEN2/PEN2’ near the center are not bound by the OBD from the bound LT dimer, probably because the linker to the helicase domain anchored to the AT-rich origin is too short for the OBD to reach PEN2. Dimerization of LT is not through the ODB, but through the helicase domains. The H513 of the β-hairpin (β-HP) and R456/F459 of the DRF-loop contacting the oriDNA are shown in the boxed inset. The oriDNA is not distorted or meltedin this intermediate complex. (**B**) Assembly of two head-head hexamers from the dimer intermediate in (**A**), which forms a near-planar closed-ring instead of the lock-washer open-ring, as predicted based on the hexamer-oriDNA structure here and the prior EM studies (Cuesta et al., 2010; Valle et al., 2006). The origin sequences at the bottom are aligned to the known binding locations on the LT double hexamer, in which the AT-rich sequences of the AT/EP halves are bound by the helicase domain. Red stars indicate the melted/distorted AT-rich sequences as identified biochemically upon assembly of LT double hexamer in the presence of ATP (Borowiec et al., 1990; Borowiec and Hurwitz, 1988). The same studies also showed that the melting of the AT-half origin is much less extensive if ADP was used instead of ATP, even though both ADP and ATP induced similar melting on the EP-half origin. Green stars indicate the melted/distorted sequence in the co-crystal structure of the ADP-bound LT hexamer in complex with the AT-half origin (with the two smaller stars indicating less distortion). It is expected that when the changes in LT conformation are coupled to the binding/hydrolysis of cyclic ATP, the extensively melted/distorted oriDNA will be propagated to form a pair of replication forks and thus to initiate DNA replication. **DOI:** http://dx.doi.org/10.7554/eLife.18129.013

**Figure 5—figure supplement 1.** The alignment of the structures of SV40-origin DNA bound to OBD alone (LT131-259) and to the OBD-helicase domain (LT131-627) of LT. The alignment is based on the origin DNA sequences in the structures with the 64-bp core origin sequence shown at the top. (**A**) The full core origin sequence of SV40. The EP-half (left) and AT-half (right) origin are capable of supporting hexamer assembly. The four PENs (in red and pink) and the newly identified pseudo-PEN (in blue) are recognized by OBD. The AT-rich sequence interacts with the helicase domain. (**B**) Structures of the four PENs bound by individual OBDs, (**C**) the full EP-half origin bound by dimeric LT131-627, and (D) the full AT-half origin bound by hexameric LT131-627. For comparison between the dimeric and hexameric LT131-627, the EP-half origin bound to the dimeric LT131-627 is aligned to the right side with the AT-half. LT131-627 (containing the OBD-helicase domain) is capable of forming a hexamer on each half origin and a double hexamer on a full-origin. Note that when a full hexamer is assembled on each half origin, only the helicase domain hexamerizes, the six OBDs are disordered in the structure, possibly because of the dynamic competition for binding to the three available binding sites (two PENs and one pseudo-PEN). When the LT131-627 dimer is bound to an half origin, only the helicase domain dimerizes, and the two OBD domains that are bound to PEN1 and pseudo-PEN separately, with an 180° inversion, do not interact with each other. **DOI:** http://dx.doi.org/10.7554/eLife.18129.014

Biochemistry studies have shown that the melting of the EP- and AT- halves of the origin can be induced by the assembly of LT onto the origin dsDNA in the presence of ATP or ADP, without the need for ATP hydrolysis (Borowiec and Hurwitz, 1988). Interestingly, even though the melting of the EP-half origin is similar in the presence of ATP or ADP, the melting of the AT-half origin is much less profound with ADP than it is with ATP (Borowiec and Hurwitz, 1988), indicating the intrinsic differences in melting between the two halves of the origin. The LT-origin dsDNA complex structure presented here corroborates these biochemical studies and provides direct structural data showing the locally melted region of the AT-half of the origin with ADP binding. We were never able to obtain dsDNA co-crystals in the presence of ATP, and so we were unable to compare AT-half origin melting with ATP versus that with ADP binding at a structural level. Because a previous report showed that the ATP-bound LT hexamer has a central channel that is about 3–5 Å narrower than the ADP-bound hexamer (Gai et al., 2004b), it is conceivable that ATP-binding would generate more extensive melting of the AT-rich origin. We did obtain co-crystals of hexameric LT with the EP-half origin dsDNA, but the diffraction quality was poor and we were unable to obtain high-resolution structural data to describe the melting EP-half in order to compare the intrinsic differences between the EP- and AT- halves of the origin in terms of hexamer formation and the associated remodeling of the origin.

### The assembly path of a LT hexamer/double hexamer on origin DNA

With the co-crystal structures of the LT dimer bound to the EP-half origin and the hexamer bound to the AT-half origin determined to date, we can begin to postulate a pathway for LT assembly at the origin (Figure 5). At the initial stage of LT assembly, a LT dimer binds to each half of the origin through initial OBD interactions with PEN1 and a newly identified pseudo-PEN site (Figure 5A). This allows the AAA+ domain to contact, via β-hairpin and DRF loop residues, the AT-rich sequences of the AT- and EP-halves of the origin through charge and DNA shape readouts (Figure 5A inset) (Chang et al., 2013). The importance of this interaction of origin DNA with β-hairpin residues H513 and K512 is consistent with previous studies showing that mutations in these residues abolish origin melting by LT (Kumar et al., 2007). Furthermore, mutations of the E1 helicase equivalent His residue, H507 of E1, also abolish origin melting by E1 (Liu et al., 2007; Schuck and Stenlund, 2011). Even though no stable trimer or tetramer intermediates of LT-oriDNA were observed, the formation of the stable LT dimer-oriDNA intermediate complex does not cause origin DNA distortion or melting (Chang et al., 2013). Interestingly, previous biochemical evidence has suggested that E1 helicase formed a trimer intermediate complex instead of a dimer on each half of the origin DNA, which melts the origin DNA before hexamer/double hexamer formation (Liu et al., 2007).

The LT dimer-oriDNA intermediate complex formed on the AT- and EP-halves of the origin can then act as a nucleation event that recruits new subunits to form the ring-shaped hexamer/double hexamer around the oriDNA (Figure 5B). The helicase domains of each hexamer then bind to the AT-rich sequences, while the six OBDs take on dynamic conformations, loosely interacting with the limited number of PEN/pseudo-PEN sites. Upon completion of LT hexamer/double hexamer assembly, the helicase domains of the six LT subunits form a tight, near-planar ring, rather than a spiral conformation, around the dsDNA. Concurrent with the assembly of this ring with a narrow central channel around the AT-rich sequences , local origin melting within the helicase domain may be achieved as a result of the formation of the narrow channel, which consists of the β-hairpins and DRF loops. The narrow channel compresses (or squeezes) the two phosphate backbones of the dsDNA to distort and melt the origin DNA. It is possible that more helical subunits are added to adimer intermediate, which converts to a planar arrangement once a full hexamer is formed, a process that could provide further energy for distorting/melting the oriDNA.

Models with spiral assembly by LT have been proposed previously (Bochkareva et al., 2006; Meinke et al., 2007); in these models, which are based on structural studies using OBD alone binding to its PEN (GAGGC) recognition sequence, propose that the OBD domain assembles into a spiral conformation. Several co-crystal studies of the isolated OBD domain of LT (or E1) have revealed how individual OBD recognizes the PEN DNA sequences (Bochkareva et al., 2006; Enemark et al., 2002; Meinke et al., 2007; Meinke et al., 2013): individual OBDs do not interact with each other, but bind tightly to the PENs using the same interactions (Figure 5—figure supplement 1A,B). However, the OBDs in the hexameric LT131-oriDNA complex structure do not bind to the PENs and are disordered (Figure 5—figure supplement 1D). The disordered OBDs in the hexamer complex also differ from the well-ordered OBDs of the LT131 dimer-oriDNA complex (Chang et al., 2013), in which one OBD (OBD1) binds to PEN1 and the other OBD (OBD2) bind to a pseudo-PEN site with about 180° rotation (Figure 1—figure supplement 1B, Figure 5—figure supplement 1C), with no interactions between the two OBDs. However, the helicase domains of the same two LT molecules bind to the AT-rich oriDNA as a tight dimer with about 60° rotation to each other. This structure of LT131 dimer-oriDNA suggests that, when OBD is linked to the helicase domain, the binding of two OBDs to PEN/pseudo-PEN probably functions to coordinate with the binding of the helicase domain to the AT-rich sequences where the initial melting occurs. Furthermore, when a complete closed hexameric ring is assembled around each half origin, it creates a problem of six OBDs with only three available binding sites (PEN1, PEN2 and one pseudo-PEN). The disordered OBDs in the hexamer-oriDNA structure indicate that OBD1 and OBD2 of the initial dimer-oriDNA intermediate no longer bind to oriDNA tightly, probably because of competition for limited binding sites among the six OBDs. This provides an explanation for the lack of well-defined electron density for the six OBDs in the hexamer structure, which is also consistent with our prior low-resolution EM studies showing the flexibility of the OBDs in the central part of the double hexamer structure (Cuesta et al., 2010; Valle et al., 2006).

In summary, the complex structure of the LT hexamer assembled on its partially melted origin dsDNA provides the first view of the detailed atomic interactions between a hexameric initiator/helicase and oriDNA, and yields novel insights into a possible mechanism of origin melting. To convert this partially melted origin to a fully opened origin, represented by a pair of replication forks, the melted ssDNA must find a way to exit the hexameric channel, as LT has been shown to translocate preferentially along one ssDNA during unwinding (Yardimci et al., 2012) and E1 has been shown to bind ssDNA (Enemark and Joshua-Tor, 2006). But LT unwinding activity can bypass a polypeptide road-block (similar to the size of a ssDNA) cross-linked to DNA substrates, suggesting that LT hexamers have sufficient plasticity to alter their conformation around DNA and allow the passage of ssDNA without falling apart (Yardimci et al., 2012). At present, we have no data regarding this process that might reveal how the initial melting of oriDNA propagates into fully open replication forks. Nevertheless, the partially melted AT-half origin within the LT helicase channel may represent a snapshot of the initially melted origin primed for further propagation into two bi-directional forks in the SV40 viral replication system and in other related eukaryotic replicons.

## Materials and methods

### Cloning, expression, and purification of LT

LT construct 131–627 (LT131) (Figure 1A) was cloned in a pGEX-6p-1 vector as a GST fusion to the N-terminus of LT. The LT protein was purified as previously described (Greenleaf et al., 2008). Briefly, the GST fusion protein was purified by glutathione affinity chromatography, followed by precision protease digestion to release LT from the GST. Gel filtration chromatography using Superdex-200 on FPLC was used to further purify the LT protein, which was concentrated to 10–20 mg/ml and stored at –80°C for crystallization.

### DNA preparation for co-crystallization

The AT-half origin dsDNA (Figure 1B) was prepared by annealing 5’-GGCCTCGGCC TCTGCATAAA TAAAAAAAAT TAT-3’ and 5’-TAATTTTTTT TATTTATGCA GAGGCCGAGG CCT-3’ as described below. The oligonucleotides (Operon) were purified through a Mono Q ion exchange column. The two purified oligonucleotides were mixed at a 1:1 molar ratio and annealed by heating to 90°C followed by slow cooling to room temperature over 30 min. Gel filtration chromatography using Superdex 75 was used to separate dsDNA from unannealed ssDNA. Purified dsDNA was concentrated to ~200 nM and stored at –20°C for co-crystallization.

### Helicase assay of preformed stable complex of LT with origin DNA

It was reported previously that the full length LT in a preformed complex with oriDNA is active in unwinding the oriDNA (Uhlmann-Schiffler et al., 2002). In order to test whether the LT131-627 construct in a preformed complex with oriDNA is also active in unwinding oriDNA, we carried out helicase assays of the preformed LT131-oriDNA complex and the un-preformed LT131-oriDNA mixture. To obtain the preformed LT131-oriDNA complex, LT131 protein and a 146-bp dsDNA containing the SV40 core origin sequence was mixed in a buffer containing 20 mM Tris-Cl pH 7.5, 50 mM NaCl, 0.1 mM EDTA, 0.1 mg/mL BSA and 1mM DTT, and the mixture was incubated for 60 min at 20°C to allow LT to bind to the oriDNA. Then, 4 mM ATP was added to the mixture for another 30 min incubation to allow ATP binding (but no hydrolysis in the absence of Mg^2+^) locking in the LT hexamer. Such preformed LT-oriDNA complex is stable for up to six hours without obvious dissociation (Figure 1C). To start the unwinding reaction, 10 mM MgCl_2_ was added to the preformed LT131 hexamer-oriDNA complex and the mixture was incubated at 37°C for 45 min. The reaction was terminated by adding 0.1% SDS, 25mM EDTA and 10% glycerol, and the reaction mixture was analyzed on 12% native polyacrylamide gel in 1X TBE buffer. As a control, the unwinding assay was also conducted side-by-side with un-preformed LT-oriDNA complex, in which reaction cocktails missing LT and Mg^2+^ were mixed on ice right before the unwinding assay (to prevent formation of LT-oriDNA complex), with the MgCl_2_ and LT protein added last to initiate the reaction.

### Co-crystallization and data collection

LT131 was mixed with the purified AT-half or EP-half origin dsDNA at a molar ratio of 6:1 (LT monomers: dsDNA) in the presence of 1mM ADP or ATP. Crystals with the same space group and cell dimensions were obtained only in the presence of ADP using the hanging drop method in a buffer containing 70 mM Hepes pH 7, 40 mM MgCl_2_, 5 mM MnCl_2_, and 10 mM DTT at 4°C. Crystals were transferred to the same buffer with the addition of 20% MPD for flash freezing with liquid nitrogen. Crystal diffraction data were collected at synchrotron beamlines at the Lawrence Berkeley National Laboratory and Argonne National Laboratory. The datasets were processed using HKL2000; the statistics are summarized in Table 1.

### Structure determination and refinement

The initial phases of the structure were solved by molecular replacement (MR) using the LT helicase domain structure in the ADP-bound form (PDB code 1SVL) as the search model with the program PHASER, which located a hexamer in one asymmetric unit. The electron density map calculated using the MR solution model of LT revealed some DNA electron density in the central channel, which was not very well featured at this stage. We improved the electron density map through six-fold multi-domain NCS averaging (i.e. separating the helicase domain into the Zn-domain and the AAA+ domain for two-domain six-fold NCS averaging) with solvent flattening prior to any DNA model building, using the CCP4 program DMMULTI. For NCS averaging, the residues on these β-hairpins and the loops (in particular, residues 330–340 of the Zn-domain, 509–518 of the β-hairpins, and 452–463 of the DRF loop) facing the central channel were deleted from the MR model for two major purposes. The first purpose was to avoid model bias because these β-hairpin and loop residues may have different conformations due to interactions with DNA. The second purpose was to calculate a tight mask (1.0 Å radius from atoms) covering the LT model with the central residues/loops deleted for NCS averaging. This was done so that the central channel space, where the DNA is located, would be completely masked out for NCS averaging, crucial for revealing the unbiased DNA density in the NCS averaged map. The mask was smoothed and islands inside the mask were removed using program MAMA in the RAVE suite (Kleywegt and Jones, 1999). The six-fold NCS averaging (50 cycles) using the improved tight mask yielded a greatly improved electron density map in the central channel, which revealed clear base-pair steps in the helical nature of the DNA density in the central channel (Figure 2—figure supplement 1A). This NCS averaged map was used to build the model ofthe DNA and the deleted residues/loops of LT in the central channel using program 'O'. However, for the fuzzy density of the N-terminal OBD, no significant improvement was achieved. The six OBD domains were only be visible as six blobs of density at low sigma level near, but not touching, the DNA density in the center. As a result, OBDs could not be built into the structure model.

The initially built model was refined by simulated annealing using Phenix, and the refined model was used for further reiterative model building and refinement. While all 32-bp steps of the AT-half sequence were visible on the NCS averaged electron density map, we built all 32-bp, plus the two 3’-T overhang (Figure 2A,B, Figure 1—figure supplement 1C). While all the DNA base pairs show strong electron densities, the density for the phosphate backbone is weaker, possibly because of the NCS-averaging effect of the six LT subunits. All the deleted LT residues in the central channel were rebuilt back into the model. The DNA register in the final model was confirmed using Bromo-dC labeled dsDNA (Figure 2—figure supplement 1B–E). The DNA register is also consistent with both the complex structure of LT131 dimer bound to the EP-half origin (Figure 1—figure supplement 1C) (Chang et al., 2013) and the biochemistry data on origin DNA binding (Joo et al., 1998; Kim et al., 1999; Sreekumar et al., 2000). The final model containing the LT helicase domain and a 32-bp origin DNA from the LT131 construct has very good refinement and geometry statistics, as shown in Table 1.

## Additional files

Supplementary file 1. The detailed interactions between oriDNA and the Zn-domain channel of LT hexamer helicase. The oriDNA sequences interacting with the Zn-channel of LT are indicated by a black bar on the right panel. The abbreviations and signs in the summary table are as follows:Arrow → donates the interactions between the indicated LT amino acids with the specific DNA residues through the Pi (phosphate via charge or hydrogen bond) from the major groove (MaGv), minor groove (MiGv), or/and directly on the DNA backbones (BkBn). **DOI:** http://dx.doi.org/10.7554/eLife.18129.015

Supplementary file 2. Detailed interactions between oriDNA and the AAA+ domain channel of LT hexamer helicase. The oriDNA sequences interacting with the β-hairpin and DRF-loop of LT AAA+ domain are indicated by a green bar on the right panel. The abbreviations and signs in the summary table are as follows: Arrow → donates the interactions between the indicated LT amino acids with the specific DNA residues through the Pi (phosphate via charge or hydrogen bond), bs (base via hydrophobic or hydrogen bond), or bb (backbone via Van der Waals), from the major groove (MaGv), minor groove (MiGv), or/and directly on the DNA backbones (BkBn). **DOI:** http://dx.doi.org/10.7554/eLife.18129.016
